RETRACTED

# LncRNA XIST promotes the progression of laryngeal squamous cell carcinoma via sponging miR-125b-5p to modulate TRIB2

**DOI:** 10.1042/BSR20193172

**Published:** 2020-04-09

**Authors:** Chunxiu Liu, Zhenjun Lu, Hui Liu, Shenfa Zhuang, Ping Guo

**Affiliations:** 1 Department of Otolaryngology, Jining First People’s Hospital of Shandong Province, Jining, Shandong, China; 2 Department of Otolaryngology, The Third People’s Hospital, Qingdao, Shandong, China

**Keywords:** laryngeal squamous cell carcinoma, LncRNA XIST, miR-125b-5p, TRIB2

## Abstract

**Objective:** X inactivate-specific transcript (XIST) is an attractive long noncoding RNA (lncRNA) functioning as an indicator of various human tumors, including laryngeal squamous cell carcinoma (LSCC). The present study was conducted to explore a novel regulatory network of lncRNA XIST in LSCC cells.

**Materials and methods:** Quantitative real-time polymerase chain reaction (QRT-PCR) was used to detect the expression levels of XIST, miR-125b-5p and TRIB2 in LSCC cells and tissues. Cell proliferation, apoptosis, migration and invasion were detected by Cell Counting Kit-8 (CCK-8), flow cytometry and Transwell assays, separately. The relationship among XIST, miR-125b-5p and tribbles homolog 2 (TRIB2) was predicted by starBase v2.0 or TargetScan and confirmed by Dual-luciferase reporter assay. The TRIB2 protein expression was quantified by Western blot assay. Murine xenograft model was utilized to validate the role of XIST *in vivo*.

**Results:** XIST was notably up-regulated in LSCC tissues and cells, and the high level of XIST was associated with the low survival rate of LSCC patients. XIST knockdown markedly repressed cell proliferation, migration and invasion and promoted the apoptosis of LSCC cells and the effects were antagonized by loss of miR-125b-5p. MiR-125b-5p was a target of XIST in LSCC cells, and it could bind to TRIB2 as well. Moreover, XIST-loss-induced down-regulation of TRIB2 could be significantly reversed by miR-125b-5p knockdown. XIST promoted the growth of LSCC tumor *in vivo*.

**Conclusion:** LncRNA XIST promoted the malignance of LSCC cells partly through competitively binding to miR-125b-5p, which in turn increased TRIB2 expression.

## Introduction

Laryngeal cancer is the second-highest incidence of squamous cell carcinoma (SCC) in otolaryngology, head and neck surgery [1,2]. Laryngeal squamous cell carcinoma (LSCC) accounts for approximately 95% pathological type of laryngeal cancer, with increasing incidence rate in the past decades [3]. Breathing, pronunciation and swallowing are the main physiological functions of the larynx, so laryngeal cancer was usually associated with the high morbidity and mortality, despite amounts of efforts have been made for laryngeal cancer treatment [4]. Accordingly, it becomes necessary to explore more scientific and rational comprehensive treatment through finding new biological indicators which were related to prognosis and diagnosis of patients with LSCC.

RETRACTED

The long non-coding RNAs (lncRNAs) were identified as key *cis*- or *trans*-regulators of gene expression with the length exceeding 200 nucleotides and participated in pathological process of human carcinoma including LSCC [5,6]. X inactivate-specific transcript (XIST), a novel X inactivation center (XIC)-located lncRNA, might alternate heterochromatin stability leading to changes in gene expression thereby to impact cancer malignant progression [7]. XIST-induced chromosome inactivation was related to a selective disadvantage in fibrosarcoma cells [8]. Meanwhile, previous studies suggested that XIST overexpression was highly correlated with poor prognosis of patients with various cancers, such as breast cancer [9], pancreatic cancer (PC) [10] and brain cancer [11]. Nevertheless, the function of XIST in LSCC has not been fully elucidated.

Recent studies revealed numerous microRNAs (miRNAs) were involved in tumor process as targets of lncRNAs. In osteosarcoma (OA), not only miR-1277-5p but also miR-137 was identified as binding targets of lncRNA XIST and they were low-expressed in OA tissues and cells [12,13]. Shen et al*.* also reported that epithelial–mesenchymal transition (EMT) capacity was restrained by XIST-loss-induced miR-429 up-regulation in PC cells [14]. Previous studies demonstrated that miR-125b-5p was notably down-regulated in esophageal squamous cell carcinoma (ESCC) and negatively regulated HMGA2 expression [15]. Other investigators discovered that miR-125b-5p was a potential biomarker of LSCC [16]. However, the potential regulatory role of miR-125b-5p and its association with XIST in LSCC have been rarely reported in LSCC.

The kinase-like protein tribbles homolog 2 (TRIB2) was implicated in the survival of liver cancer cells as an important regulator of the Wnt signaling pathway [17]. Overexpression of TRIB2 also existed in acute myeloid leukemia (AML) cells and TRIB2 functioned as an oncogene via regulating C/EBPα and E2F1 repression [18]. Histological study of TRIB2 in colorectal cancer demonstrated that up-regulation of miR-511 or miR-1297 contributed to TRIB2-inhibition-induced cell proliferation arrest in lung adenocarcinoma cells [19]. Given much importance of TRIB2 in cancer progression, it is meaningful to explore its potential role in LSCC.

In our study, we explored XIST expression in LSCC cells and tissues and its functional role in cell proliferation, anti-apoptosis, migration and invasion of LSCC cells. Meanwhile, the correlation among XIST, miR-125b-5p and TRIB2 was uncovered, which might provide a promising molecular target for XIST/miR-125b-5p/TRIB2 axis-associated LSCC treatment.

RETRACTED

## Materials and methods

### Ethics statement and tissue acquisition

Ethical issues, relating to cancer tissues and matched normal tissues, were supervised by the Ethics Committee of Jining First People’s Hospital of Shandong Province. The laryngeal cancer tissues were obtained from 40 patients who underwent surgery at Jining First People’s Hospital of Shandong Province and signed informed consents before and tissues were immediately preserved at −80°C. The animal work was taken place in Jining First People’s Hospital of Shandong Province, and we used 2% methoxyflurane in the experiment work for euthanasia of the mouse, which was in accordance with the National Institutes of Health.

### Cell culture and transfection

LSCC cell lines (AMC-HN-8 and M4E cells) and nasopharyngeal epithelial cells (NP69 cells) were obtained from the Cell Bank, China Academy of Sciences (Shanghai, China) and incubated in Dulbecco’s modified Eagle’s medium (DMEM; Invitrogen, Carlsbad, CA, U.S.A.) including 10% fetal bovine serum (FBS; Invitrogen) at 37°C with 5% CO_2_ and humidified air. Vectors or oligonucleotides (including small interference RNA (siRNA) against XIST (si-XIST), has-miR-125b-5p mimic/inhibitor, pcDNA-TRIB2 vector and each matched controls) were constructed by GenePharma (Shanghai, China) and transfected into AMC-HN-8 and M4E cells, applying Lipofectamine® 2000 reagent (Invitrogen). The specific transfection steps referred to the instruction manual. At 48 h post transfection, cells were harvested for subsequent analyses.

### RNA isolation and quantitative reverse transcription polymerase (qRT-PCR)

TRIzol Reagent ((Invitrogen) and chloroform were used to isolate total RNA of LSCC tissues or cells, and then the total RNA was precipitated with iso-propanol (VWR International). The RNA precipitation was purified by 70% ethanol and air-dried and then resuspended in sterile water (without nuclease). The concentration of total RNA was detected by an Eon™ Microplate Spectrophotometer (BioTek Instruments, Inc., Winooski, VT). One Step PrimeScript miRNA cDNA synthesis kit (Takara Bio Inc., Dalian, China) was used to carry out the reverse transcription reaction. SYBR® Premix Ex Taq™ II (Takara) was used for PCR on a MiniOpticon™ (Bio Rad, Hercules, CA, U.S.A.). 2^−ΔΔCT^ method was used to calculate the levels of XIST, miR-125b-5p and TRIB2, normalized to U6 small nuclear RNA (U6-snRNA) and housekeeping gene glyceraldehyde-3-phosphate dehydrogenase (GAPDH), separately. The PCR condition was listed as below: denaturation (30 s, 94°C), annealing (30 s, 58°C) and extension (30 s, 72°C, 30 cycles). The involved primer sequences were as follows: XIST, forward 5′- GCATAACTCGGCTTAGGGCT-3′, reverse 5′-TCCTCTGCCTGACCTGCTAT-3′; miR-125b-5p, forward 5′-TCCCTGAGACCCTAACTTGTGA-3′, reverse 5′-AGTCTCAGGGTCCGAGGTATTC-3′; TRIB2, forward 5′-CACAGGTCTACCCCCATCAC-3′, reverse 5′-CCCGATACAAGAAACGCAAT-3′; GAPDH, forward 5′-CCAAAATCAGATGGGGCAATGCTGG-3′, reverse 5′-TGATGGCATGGACTGTGGTCATTCA-3′; U6, forward 5′-CTCGCTTCGGCAGCACA-3′, reverse 5′-AACGCTTCACGAATTTGCGT-3′.

RETRACTED

### Cell counting Kit-8 (CCK-8) assay

Transfected cells (2.5 × 10^3^ cells/100 µl/well) were prepared for proliferation assay and seeded into 96-well plates. Cells were respectively cultured for 24, 48 and 72 h until 10 µl CCK-8 regent (DOJINDO, Kumamoto, Japan) was separately added into each well for another 4 h. A microplate reader (Bio-Rad, Hercules, CA, U.S.A.) was used to test the optical density (OD value) at an absorbance of 450 nm.

### Flow cytometry assay

Annexin V-fluorescein isothiocyanate (FITC)/propidium iodide (PI) Apoptosis Detection Kit (Immunotech, Marseille, France) was used for cell apoptosis assay. All experimental cells were collected and the concentration was adjusted to 1 × 10^6^ cells/ml. About 200 µl cell suspension was used for assay and was re-suspended in 300 µl binding buffer and gently mixed with 5 µl Annexin V-FITC/PI for 15 min in the dark. FACScan flow cytometer (Becton Dickinson, San Jose, CA, U.S.A.) was used for analysis of apoptosis rate.

### Transwell assay

Transfected cells were incubated with serum-free DMEM for 12 h until Transwell assay. Matrigel (Corning Life Sciences, Corning, NY, U.S.A.) was stored at 4°C overnight for preparation. The Transwell chambers were placed into each well of 24 well-plate, respectively. DMEM (500 µl; containing 20% FBS) was added into each lower chamber; meanwhile, transfected cells, at the concentration of 1 × 10^5^ cells/100 µl/well (using serum-free DMEM), were seeded into the upper chambers for migration test or into the upper chamber already coated with 10 µl Matrigel for invasion test. After 48-h conventional incubation, Transwell chambers were taken out and the inner cells were lightly wiped off and then put into a new 24 well-plate with 4% paraformaldehyde (600 µl). Until fixed for 5 min, cells were stained with 0.1% Crystal Violet for 10 min. Finally, cells were calculated in five random fields under an inverted microscope.

### Dual-luciferase reporter assay

The sequence of XIST or TRIB2 was synthesized and cloned into the pGL3 Dual-luciferase reporter vector (Promega, Madison, MI, U.S.A.). The generated new reporter vectors were named as pGL3-XIST-WT (wild-type of XIST), pGL3-XIST-Mut (mutant-type of XIST), pGL3-TRIB2-WT (wild-type of TRIB2) and pGL3-TRIB2-Mut (mutant-type of TRIB2), respectively. The pGL3-XIST-WT and pGL3-TRIB2-WT contained the predicted binding sites of miR-125b-5p. Above reporter vectors were co-transfected into AMC-HN-8 and M4E cells with miR-NC or miR-125b-5p mimic using Lipofectamine® 2000. After 48 h, the relative luciferase activity was examined using a Dual-luciferase Reporter Assay kit (Promega), normalized to that of Renilla.

RETRACTED

### Western blot analysis

RIPA lysate was added into tissues or cells to extract proteins and the concentration of the total proteins was quantified by the bicinchoninic acid (BCA) method using a BCA-kit (Pierce Biotechnology, Inc., Rockford, IL, U.S.A.). Sodium dodecyl sulfate polyacrylamide gel electrophoresis (SDS-PAGE) was used for the isolation of target proteins and then separated proteins were transferred onto polyvinylidene difluoride (PVDF) membranes (Millipore, Bradford, MA, U.S.A.) under a constant current of 1–1.5 mA/cm^2^. All membranes were dipped into 5% skimmed milk powder for 2 h, at room temperature, and immerged into diluted primary antibodies against TRIB2 or β-actin overnight at 4°C. After being washed twice with Phosphate Buffered Saline and Tween 20 (PBST), the membranes were successively incubated with horseradish peroxidase-labeled goat anti-rabbit secondary antibody for 1 h, 37°C. Above antibodies were obtained from Santa Cruz Biotechnology, Inc. (Santa Cruz, CA, U.S.A.). In the gel imager (Bio-Rad), the electrochemiluminescence (ECL; Pierce) was added dropwise to cover the hybridization membranes for photographing. Finally, the strips were analyzed using Quantity One software.

### Tumor formation in nude mice

The procedure in this experiment had gotten the permission of the Institutional Animal Care and Use Committee of Jining First People’s Hospital. The nude mice (Shanghai SLAC Laboratory Animal, Shanghai, China) were injected with AMC-HN-8 cells expressing sh-NC or sh-XIST. The volume was measured every 7 d, and the weight of LSCC tumors was measured following injection for 35 d. The tumor tissues were used for the detection of the expression of XIST, miR-125b-5p and TRIB2.

### Statistical analysis

SPSS software v.19.0 and GraphPad Prism software v.5.0 were used for data analysis. Data were expressed as mean ± standard deviation (SD), obtained from at least three independent experiments. Five-year overall survival rate was analyzed by Kaplan–Meier method. Student’s *t-*test or ANOVA was applied to assess the statistical significance, which was taken as *P* < 0.05.

RETRACTED

## Results

### Overexpression of XIST indicated poor prognosis of patients with laryngeal squamous cell carcinoma (LSCC)

Firstly, qRT-PCR was used to assess XIST expression in 40 pairs of LSCC tissues and matched adjacent normal tissues. As shown in Figure 1A, XIST was obviously up-regulated in LSCC tissues compared with that in adjacent normal tissues. Further, analysis of 5-year overall survival rate by Kaplan–Meier method revealed that high level XIST was correlated with low survival rate (*P* = 0.0423) (Figure 1B). The expression of XIST was positively correlated with tumor size, TNM stage, tumor differentiation and metastasis of LSCC patients (Table 1). LSCC cell lines (AMC-HN-8 and M4E cells) and nasopharyngeal epithelial cells (NP69 cells) were also chosen for examination of XIST expression. The data of qRT-PCR analysis proved higher level of XIST existed in LSCC cells, compared with NP69 cells (Figure 1C). In a word, we found that XIST, as an oncogene in LSCC, could be a potential predictor of cancer development.

**Figure 1:** XIST expression in LSCC cells or tissues and its association with 5-year overall survival rate were assessed Notes: (**A**) XIST expression in LSCC tissues and matched normal tissues was detected by qRT-PCR (*n*= 40). (**B**) Correlation between XIST expression and prognosis of patients with LSCC was analyzed. (**C**) QRT-PCR analysis of XIST expression was performed in LSCC cells (AMC-HN-8 and M4E cells) and nasopharyngeal epithelial cells (NP69 cells); *P <0.05.

**Table 1:** Correlation between clinicopathological characteristics and XIST expression levels in laryngeal squamous cell carcinoma patients

Characteristics	*n*	XIST		*P*
		High	Low	
Gender				
Male	19	6	13	0.906
Female	21	7	14	
Age(years)				
≥50	22	14	8	0.225
<50	18	8	10	
Tumor size				
≥3 cm	20	17	3	0.018
<3 cm	20	10	10	
TNM stage				
I+II	22	18	4	0.005
III+IV	18	7	11	
Tumor differentiation				
Moderate-high	21	14	7	0.027
Low	19	6	13	
Metastasis				
Yes	22	15	7	0.011
No	18	5	13	

### Interfering of XIST expression arrested proliferation, migration and invasion, and induced cells apoptosis in LSCC cells

Next, functional experiments were conducted to explore functions of XIST in LSCC cells. The loss of XIST was performed by transfecting small interfering RNA targeting XIST into AMC-HN-8 and M4E cells for 48 h. The result of qRT-PCR indicated that XIST expression was distinctly down-regulated in LSCC cells (Figure 2A,B). Then, cell proliferation arrest was detected in AMC-HN-8 and M4E cells with XIST suppression (Figure 2C,D). The results of flow cytometry assay demonstrated that cell apoptosis was promoted by the intervention of XIST (Figure 2E,F). Furthermore, cell migration and invasion were declined with XIST knockdown in AMC-HN-8 and M4E cells (Figure 2G,H). On the whole, XIST played an oncogenic role in LSCC through inhibiting the apoptosis while promoting the proliferation and metastasis of LSCC cells.

RETRACTED

**Figure 2:** Knockdown of XIST restrained cell proliferation and migration and invasion while induced apoptosis in LSCC cells Notes: (**A** and** B**) Si-NC or si-XIST was transfected into AMC-HN-8 and M4E cells, and the interference effects were detected by qRT-PCR at 48 h post transfection. (**C** and **D**) Cell proliferation was examined by CCK-8 assay and (**E** and **F**) flow cytometry was used to detect cell apoptosis. (**G** and **H**) Transwell assay was conducted to measure migration and invasion of transfected cells; *P <0.05.

### XIST sponged miR-125b-5p in LSCC cells

As depicted in Figure 3A, there existed complementary sites between miR-125b-5p and XIST. To explore whether miR-125b-5p was a target of XIST, Dual-luciferase reporter assay was conducted by co-transfecting wild-type and mutant form of XIST (XIST-WT and XIST-Mut) with miR-NC or miR-125b-5p mimic into AMC-HN-8 and M4E cells, separately. The luciferase activity was significantly declined in AMC-HN-8 and M4E cells co-transfected with XIST-WT and miR-125b-5p, but no difference occurred in other groups (Figure 3B,C). Then the regulatory relationship between miR-125b-5p and XIST was further explored in LSCC cells by transfection of si-XIST. The expression of miR-125b-5p was markedly increased by the loss of XIST in AMC-HN-8 and M4E cells (Figure 3D,E). And then, we found that the level of miR-125b-5p was lower in LSCC cells and tissues (Figure 3F,G). In general, miR-125b-5p might be a potential tumor suppressor, which was negatively regulated by XIST.

**Figure 3:** XIST sponged miR-125b-5p in LSCC cells Notes: (**A**) The binding site alignment of miR-125b-5p was predicted in XIST. (**B** and **C**) Luciferase activity was measured by Dual-luciferase reporter assay in cells co-transfected with pGL3-XIST-Wt or pGL3-XIST-Mut vectors and miR-NC or miR-125b-5p. (**D** and** E**) The relationship between miR-125b-5p and XIST was detected by qRT-PCR in LSCC cells. (**F** and** G**) The relative expression of miR-125b-5p was examined by qRT-PCR in LSCC cells and tissues (*n*= 40); *P <0.05.

### Down-regulation of miR-125b-5p abolished si-XIST-mediated effects on LSCC cells

The regulatory role of miR-125b-5p in XIST expression was further confirmed in AMC-HN-8 and M4E cells by transfection of si-XIST with or without anti-miR-125b-5p. The qRT-PCR results indicated that miR-125b-5p expression was notably elevated in AMC-HN-8 and M4E cells with loss of XIST, but this phenomenon was obviously overturned by the introduction of anti-miR-125b-5p (Figure 4A,B). Meanwhile, cell proliferation was inhibited in AMC-HN-8 and M4E cells by the transfection of si-XIST, whereas knockdown of miR-125b-5p coupled with XIST down-regulation could abolish si-XIST-mediated cell proliferation arrest (Figure 4C,D). Flow cytometry assay demonstrated that anti-miR-125b-5preversed the promoting effect of XIST interference on the apoptosis of LSCC cells (Figure 4E,F; Supplementary Figure S1A,B). Similarly, the inhibition of migration and invasion in LSCC cells with XIST loss was restored by knockdown of miR-125b-5p (Figure 4G,H; Supplementary Figure S1C,D). All data elucidated that XIST accelerated the progression of LSCC via inhibiting miR-125b-5p.

RETRACTED

**Figure 4:** Anti-miR-125b-5p reversed the effect of XIST loss in AMC-HN-8 and M4E cells Notes: AMC-HN-8 and M4E cells transfected with si-NC, si-XIST, si-XIST+anti-miR-NC or si-XIST+anti-miR-125b-5p were classified as four groups, respectively. (**A** and** B**) QRT-PCR was used to quantify miR-125b-5p expression in the above four groups. (**C** and **D**) Cell proliferation was examined by CCK-8 assay. (**E** and** F**) By flow cytometry assay, the apoptosis rate of cells was detected in four groups. (**G** and **H**) Analysis of cell migration and invasion in four groups was conducted by Transwell assay; *P <0.05

### MiR-125b-5p was a target of TRIB2 in LSCC cells

It was predicted that hsa-miR-125b-5p bound to 3′UTR of TRIB2 (Figure 5A) by TargetScan online software. Then, the wild-type or mutant type of TRIB2 reporter vector named pGL3-TRIB2-3′UTR-WT or pGL3-TRIB2-3′UTR-Mut was transfected into AMC-HN-8 and M4E cells, along with miR-NC or miR-125b-5p mimic to explore the adhesion of miR-125b-5p on TRIB2. As shown in Figure 5B,C, the luciferase activity was markedly decreased in cells treated with TRIB2-WT and miR-125b-5p, compared with cells treated with miR-125b-5p and TRIB2-Mut. Accordingly, it was found that overexpression of miR-125b-5p could effectively repress TRIB2 expression in AMC-HN-8 and M4E cells (Figure 5D,E). In addition, the expression of TRIB2 was higher in LSCC cells (AMC-HN-8 and M4E cells) than that in nasopharyngeal epithelial cells (NP69 cells), quantified by both Western blot assay and qRT-PCR (Figure 5F). Moreover, the protein expression level of TRIB2 was elevated in LSCC tissues, compared with that in paired normal tissues, which was in accordance with the result of qRT-PCR (Figure 5G). Overall, our results demonstrated that TRIB2 expression could be directly repressed by miR-125b-5p.

RETRACTED

**Figure 5:** TRIB2 was a novel target of miR-125b-5p in LSCC cells Notes: (**A**) The potential binding sites of miR-125b-5p were predicted in 3′UTR of TRIB2. (**B** and **C**) The luciferase activity was detected in AMC-HN-8 and M4E cells transfected with pGL3-TRIB2-3′UTR-WT and pGL3-TRIB2-3′UTR-Mut reporter vectors, along with miR-125b-5p or miR-NC. (**D** and** E**) Western blot assay and qRT-PCR were used to explore TRIB2 expression in AMC-HN-8 and M4E cells with or without miR-125b-5p up-regulation. The protein and mRNA levels of TRIB2 were determined in LSCC cells and NP69 cells (**F**) as well as in LSCC tissues and paired normal tissues (**G**) (number of tissues: *n*= 3, for Western blot assay; *n*= 40, for qRT-PCR); *P <0.05.

### Overexpression of TRIB2 reversed miR-125b-5p-mediated effects on LSCC cells

In order to explore whether miR-125b-5p was a tumor inhibitor via targeting TRIB2, we divided AMC-HN-8 or M4E cells into four groups, then transfected with miR-NC, miR-125b-5p, miR-125b-5p+vector, or miR-125b-5p+TRIB2, separately. Then, Western blot assay and qRT-PCR were used to confirm that TRIB2 expression was significantly declined in miR-125b-5p group, compared with miR-NC group, while TRIB2 expression was increased in cells in miR-125b-5p+TRIB2 group cells, compared with miR- miR-125b-5p+vector group, in both AMC-HN-8 and M4E cells (Figure 6A,B). Synchronously, we found that miR-125b-5p repressed cell proliferation and induced cell apoptosis. Interestingly, these effects could be partially overturned by TRIB2 up-regulation in AMC-HN-8 and M4E cells (Figure 6C–F; Supplementary Figure S2A,B). The cell migration and invasion were remarkably suppressed in miR-125b-5p group, but the result was opposite in miR-125b-5p+TRIB2 group, detected by Transwell assay (Figure 6G,H; Supplementary Figure S2C,D). To sum up, miR-125b-5p inhibited the malignant potential of LSCC cells through suppressing TRIB2.

**Figure 6:** TRIB2 was negatively correlated with miR-125b-5p in LSCC cells Notes: MiR-NC, miR-125b-5p, miR-125b-5p+vector, or miR-125b-5p+TRIB2 vector was separately transfected into AMC-HN-8 or M4E cells as four groups. (**A** and** B**) Western blot assay and qRT-PCR was used to detect TRIB2 expression in transfected cells. (**C** and **D**) CCK-8 assay was conducted to assess cell proliferation. (**E** and **F**) The flow cytometry assay was performed to detect cell apoptosis rate in transfected cells. (**G** and **H**) The migration and invasion were assessed by Transwell assay in AMC-HN-8 and M4E cells in four groups; *P <0.05.

### Knockdown of XIST suppressed TRIB2 expression through sponging miR-126b-5p

Finally, Western blot assay and qRT-PCR were conducted to explore the underlying relationship among lncRNA XIST, miR-125b-5p and TRIB2 in LSCC cells. The mRNA expression level of TRIB2 was clearly down-regulated in AMC-HN-8 and M4E cells with XIST loss, whereas suppression of miR-125b-5p reversed the result, quantified by qRT-PCR (Figure 7A,B). Additionally, interfering XIST expression also markedly decreased the protein of TRIB2, which was reversed by miR-125b-5p repression in LSCC cells, according to the result of Western blot analysis (Figure 7C,D). Based on the above results, we discovered that lncRNA XIST down-regulation could inhibit TRIB2 expression via directly sponging miR-125b-5p in LSCC cells.

RETRACTED

**Figure 7:** The loss of XIST induced TRIB2 repression through binding to miR-125b-5p in LSCC cells Notes: (**A** and **B**) QRT-PCR was performed to quantify TRIB2 expression after si-NC, si-XIST, si-XIST+anti-miR-NC, and si-XIST+anti-miR-125b-5p were transfected into AMC-HN-8 and M4E cells for 48 h. (**C** and **D**) The protein expression level of TRIB2 was examined in the transfected cells by Western blot assay; *P <0.05.

### XIST depletion suppressed the tumor progression of LSCC *in vivo*

We validated the role of XIST through murine xenograft model *in vivo*. The volume and weight of LSCC tumors were markedly lesser in sh-XIST group in comparison with that in sh-NC group (Figure 8A,B). QRT-PCR and Western blot were performed to measure the expression of XIST, miR-125b-5p and TRIB2 in tumor samples. As shown in Figure 8C–E, the level of XIST and the RNA and protein expression of TRIB2 were decreased in sh-XIST group, while the expression of miR-125b-5p revealed an opposite phenomenon.

**Figure 8:** XIST depletion suppressed the tumor progression of LSCC *in vivo* Notes: (**A**) The volume of LSCC tumors was measured every 7 d. (**B**) The weight of LSCC tumors was detected following injection for 35 d. (**C**–**E**) The expression of XIST, miR-125b-5p and TRIB2 was determined in tumor samples through qRT-PCR and Western blot assay.

## Discussion

In the present study, we identified lncRNA XIST as a novel predictor of laryngeal squamous cell carcinomas (LSCC) and XIST overexpression was strongly correlated with poor prognosis of patients with LSCC. In the previous report, high level of XIST was quantified in LSCC *in vitro* and *in vivo*, in turn promoting tumor growth and reducing cell apoptosis rate [20]. Similar experiments were conducted on our efforts and we uncovered that XIST was markedly up-regulated in LSCC tissues (*n* = 40) and AMC-HN-8 and M4E cells. Moreover, the higher XIST expression usually represented the lower 5-year survival rate of patients with LSCC, via Kaplan–Meier analysis. These discoveries were in conformity with the report of Xiao et al*.* [21]. Additionally, silencing XIST gene slowed down cell proliferation, as well as weakened anti-apoptosis, migration and invasion abilities of LSCC cells, which further determined the promotion role of XIST in LSCC.

RETRACTED

Recently, miR-92b has been certified as a target inhibitor of XIST in hepatocellular carcinoma (HCC) [22]. Analogously, exosomal miRNA-503 was accumulated by loss of XIST resulting in tumor metastasis was repressed, which provided an attractive doctoring for breast cancer in the report of Xing et al*.* [11]. These researches manifested that miRNAs had intimate association with lncRNA XIST. MiR-125b-5p expression was increased in HCC with hepatitis B virus (HBV) infection [23]. But oppositely, reduction of miR-125b-5p was detected in LSCC cells and miR-125b-5p regulated cell glycolysis and growth by directly targeted hexokinase-2 (HK2), a key enzyme for glycolysis process [24]. Using online software, we manifested miR-125b-5p, as a target of XIST, was notably low-expressed in LSCC cells (AMC-HN-8 and M4E cells) and tissues corresponding to Lokman et al*.* [25]. The small interference XIST (si-XIST) was transfected into LSCC cells in our study, which induced obviously up-regulation of miR-125b-5p, thereby arresting LSCC cells growth and metastasis. Concurrently, anti-miR-125b-5p expression could overtly abolish the XIST-loss effect. These data indicated that the promotive action of XIST to LSCC progression exerted through directly bating miR-125b-5p expression.

Tribbles homolog 2 (TRIB2) belongs to Tribbles pseudokinases, playing a pivotal role in etiology of multifarious cancers [26,27]. Investigators found TRIB2 expression was elevated in colorectal cancer (CRC) and TRIB2 overexpression promoted cell proliferation and deferred cellular senescence of CRC partially relying on direct regulation of p21 expression and transcription factor AP4 expression [28]. In another study, promoter activity of TRIB2 might be declined in miR-206/miR-140-elevated lung adenocarcinoma cell, weakening cell invasive ability and proliferation [29]. We found that has-miR-125b-5p bound to 3′UTR of TRIB2 and the low-expression of TRIB2 was detected in LSCC cells with up-regulated miR-125b-5p expression. In addition, high mRNA and protein expression of TRIB2 existed in LSCC cells and tissues. The similar effect of TRIB2 in cervical cancer was uncovered by Xin et al*.* [30]. Furthermore, the results of our rescue experiments demonstrated that up-regulation of TRIB2 reversely adjusted the inhibitive effect of miR-125b-5p overexpression on proliferation, anti-apoptosis and metastasis in LSCC cells. Mechanistically, TRIB2 expression was distinctly down-regulated in cells treated with si-XIST, whereas loss of miR-125b-5p evidently abolished the effect. Moreover, the oncogenic role of XIST was also verified through murine xenograft model. Thus, these results revealed that silencing XIST down-regulated TRIB2 expression through sponging miR-125b-5p in LSCC cells. However, due to practical limitations, we will complete related *in vivo* experiments in the future.

RETRACTED

## Conclusion

In the present study, overexpression of both lncRNA XIST and TRIB and down-regulation of miR-125b-5p were uncovered in LSCC tissues and cells. The high-level XIST usually denoted poor prognosis of patients with LSCC. XIST suppression slowed down cell growth and weakened cell metastasis and anti-apoptosis. Both XIST and TRIB2 contained the binding sites of miR-125b-5p, which was firstly predicted in our study. Reduction of XIST notably increased miR-125b-5p expression and up-regulation of miR-125b-5p reversed XIST-loss-mediated inhibitive effect on LSCC cells. On the other hand, miR-125b-5p negatively regulated TRIB2 and reversed the promotive action of XIST on TRIB2 expression in LSCC cells. Our results provided a compelling XIST-miR-125b-5p-TRIB2-correlated therapy for LSCC.

## Highlights

- Both lncRNA XIST and TRIB were overexpressed in laryngeal squamous cell carcinoma (LSCC) tissues and cells, while miR-125b-5p was down-regulated.
- It was first proved that XIST acted as a novel sponge of miR-125b-5p that simultaneously targeted TRIB2.
- Knockdown of XIST overtly repressed cell proliferation, migration and invasion and increased apoptosis in LSCC cells and the effects were revered by miR-125b-5p down-regulation.

## Supplementary Material

Supplementary Figures S1-S2

## Data Availability

The analyzed data sets generated during the present study are available from the corresponding author on reasonable request.

## Abbreviations

CCK-8: Cell Counting Kit-8
CRC: colorectal cancer
HK2: hexokinase-2
lncRNA: long noncoding RNA
LSCC: laryngeal squamous cell carcinoma
QRT-PCR: quantitative real-time polymerase chain reaction
SCC: squamous cell carcinoma
si-XIST: small interference XIST
TRIB2: tribbles homolog 2
XIST: X inactivate-specific transcript
